The article "Application of Unsupervised Migration Method Based on Deep Learning Model in Basketball Training" was retracted in 2023. Reasons: unreliable results or conclusions; concerns about the data; concerns about the results or conclusions; concerns about the peer review.

# Application of Unsupervised Migration Method Based on Deep Learning Model in Basketball Training

**DOI:** 10.1155/2022/6711331

**Published:** 2022-02-23

**Authors:** Hui Sun, Yu Wang, Yujue Wang

**Affiliations:** ^1^Physical Education Department, Dongguan City College, Dongguan 523419, Guangdong, China; ^2^School of Physical Education & Sports Science, South China Normal University, Guangzhou 510006, Guangdong, China

## Abstract

Nowadays, China's sports industry has attained effective development, but the athlete's efficiency in the training process is too complex to have a scientific guarantee. Machine learning technology's help in guiding the sports training process has become a hot spot. In this work, we investigate the use of deep learning in real-time analysis of basketball sports data, utilizing research approaches such as scientific reporting, audio/video analysis, experimental research, and mathematical statistics. The suggested basketball stance action recognition and analysis system are made up of two pieces that are sequentially connected. The bottom-up stance estimate approach is utilized to locate the joint locations in the first segment, which is then used to extract the target's posture sequence from the video. The analyses are needed for a Support Vector Machine (SVM) algorithm based on the deep learning method of the space-time graph. The basketball activity of the set classification is recognized and extracted from the segmented stance sequence. The study used an auxiliary method, which is contrasted to standard training, in order to get higher accuracy and also correct player errors in a timely manner. The approach can help players rectify technical errors, develop muscle memory, and increase their abilities. The results revealed that the algorithm generated 97.7% accuracy in evaluating data from basketball training.

## 1. Introduction

Competition in sports is an enjoyable recreational activity based on sports regulations and is a significant component of physical exercise in general. Sports tournaments have drawn a large number of competitors and viewers since their inception because of their distinctive charm [1]. Sports tournaments are frequently scrutinized from a technical standpoint in an effort to improve the level of competitiveness within the sport in question. Aesthetic research into sports competitions is rare, and it focuses on discovering what makes sports so appealing and designing the optimal venue for sporting events. As clustering technology has progressed, academics have conducted much research on clustering algorithms. Because of the wide range of people who use the Internet, algorithms for making recommendations have been developed [2]—analyzing sports competitions using methods related to data mining. With such a large number of athletes and a complicated and changing sporting environment, data mining can help address the challenges encountered by sports competitions [3]. It is possible to see if previously taught or newly acquired knowledge is similar, and this similarity is the basis for transfer learning [4]. Currently, it appears that most data sets are comparable, allowing migration learning to be broadly applied across a wide range of machine learning domains. Usually, convolutional neural networks are not trained from scratch since, even with strong hardware performance, training the model takes a long time as the dataset size increases [5]. Thus, the issue of lengthy training is avoided. Using migration learning can reduce model training costs, enhance model training efficiency, and even better, maximize all of these things at the same time. Theoretically, migration learning can be used successfully in any relevant field [6]. It is important to note, however, that if there is a lack of similarity between the models to be trained and those that have already been trained, the end results will be subpar or even show negative migration [7]. Data points are grouped together as part of a machine learning approach known as clustering. Using a clustering technique, we can categorize a collection of data points into smaller groups. One characteristic should be shared by all members of a group, while the other characteristics should be wildly different. Clustering is an unsupervised learning tool and a common statistical data analysis approach in many fields. Clustering analysis is a powerful tool in data science that can help us learn more about our data. With an increased focus on improving and optimizing decision tree techniques to improve classification accuracy, application effects, and the advancement of the choice pruning process to improve decision tree algorithms' comprehensive application impact, research into decision tree algorithms is exploding right now. When a computer learns from its data, it can then use that knowledge to make predictions about the future [8]. In this technique, machines can study large-dimensional data or be relentless, similar to how humans learn. This paper evaluates the effects of sports training using an unsupervised deep learning algorithm. The following is the paper's contribution:

1. Perception analysis is used to investigate the reference image captured or retrieved from image sequences of a recorded basketball game.
2. The picture is segmented and image features extracted to undertake motion capture using a variety of image processing methods.

## 2. Related Studies

Support vector machine (SVM) is a method of unsupervised machine learning used to classify data into groups based on common characteristics. Clustering algorithms, an important area of data mining, offer a wide range of applications and are now rapidly developing [9]. Maximum edge clustering (MMC), which is based on an SVM model, according to the conclusions of the research, beats the means method. According to the conclusions of the research, clustering beats the means method [10]. XML document processing is a challenge in web data mining, as is structured text processing with structural and semantic coincidences. M&T employed the tree meta-ancestor methodology to find out what information was contained in XML documents before processing the information using methods such as clustering [11]. Because it becomes impossible to tailor decisions based on individual conditions as the number of entities grows, the response strategy and performance suffer as a result. By utilizing techniques like clustering and recommendation algorithms, we can assist specialists in making recommendations and providing coping strategies for many elements of athletes using data mining, which is uncommon in sports competitions [12].

Because of how extensively it has been studied, concepts and theories concerning sports competition have expanded to a wide range of sports. With the core and auxiliary perspectives, basketball from all angles, including the physical body and the technical and tactical skills of the players and star players, and spirit, style, and the aesthetics of the uniform and field equipment, all of which have a positive impact on our understanding of the distinctive features of basketball competition [13]. Since gradients no longer exist when the number of layers in neural networks is increased, the learning ability of neural networks can actually degrade [14]. The SVM algorithm became the de facto standard for machine learning algorithms due to its superior migration performance, which outperformed neural networks in a wide range of applications [15]. The convolutional neural network (CNN) is the first deep learning method to use a multilayer network topology in practice [16]. It reduces the number of network parameters by utilizing spatial relativity and a human visual brain structure, resulting in improved model performance [17]. By removing structural errors, good data pretreatment also makes it easier to mine the information. Individuals' periods of archery movement are not the same, and the timing at which movement techniques are applied varies at each step. When dealing with data that has a chaotic structure and a high degree of continuity, equal-width discretization works well [18].

To achieve the project's unique research objectives, association rules, clustering, and Markov-based data mining techniques have all been thoroughly explored and used in sports competitive action data mining. There are a variety of specialized data mining tools available. Because of the wide range of data mining jobs, data mining is faced with a wide range of difficult issues [19]. The most pressing problems for data mining researchers are the design of data mining languages, the use of efficient and usable data mining methodologies, and the creation of systems to create dynamic, integrated data mining environments. The conversion of kinematic data from sporting events into a standard data structure is one of the most difficult data mining issues. As sports movements vary in pace, preparation of the data is required to maintain the data's quality and structural integrity. Extensive testing and analysis are necessitated by kinematic data adaptation to data mining techniques. We look at the models discussed in the necessary references and develop our own research model based on their strengths and flaws.

Sports athlete gait identification is a hot area of research right now. Training approaches, gait identification models, and predictions of gait have all been investigated by researchers [20]. An intelligent sports training system using a combination of a convolutional neural network model and input from sensors while also controlling sports training intelligently is based on specified indicators. Using a convolutional neural network method, athletes' daily training efficiency and ability to make full use of training data have been improved. In [21], the method was proven to be useful in guiding basketball players. A convolutional neural network theory was used to investigate the diameter, weight, safety, and resistance of a sphere in sports, determining different parameters and influencing aspects of the sports training system [22]. To determine the effect of gait recognition on sports performance, neural network algorithms and other factors were combined. To show that his method is useful in improving basketball safety, the sphere's motion trajectory in conjunction with the athlete's movements has been identified. The factors that have the greatest impact on athletic training and have developed a functional relationship between gait recognition and a variety of dynamic performance using many neural network analysis approaches and chosen superresolution elements. The researchers stated sportspeople are concerned about a lack of resolution when training [23]. The multidimensional application of various data and information has been completed with numerous control experiments. A study found that employing convolutional neural networks for sports judgment was practical, even when used to improve basketball player safety under a variety of circumstances [24]. Using varied experimental data, they analyzed and evaluated the data analysis conditions needed for various sports and used convolutional neural network models to model and analyze the training process information from different sports. In order to analyze forces and evaluate the safety of multiple players' gaits in various sports based on applicable standards, researchers utilized convolutional neural network models of various athletes' gaits in various sports [25]. Data analysis in football training was carried out using the different dialectical methodology based on the convolutional neural network algorithm, and it was found to have greater advantages. Particle swarm optimization was developed to evaluate optimization at various stages after research on the influence of basketball players adopting different training methodologies and the recognition of critical training nodes. However, there is some evidence to suggest that algorithms can help athletes with dynamic movement-related gait recognition issues. The ant colony method and the particle swarm algorithm were used to build an optimization model to improve recognition accuracy for dislocation gait identification. The researchers generated an interactive 3D dynamic motion map by emulating a sports athlete's stride and correctly identifying his or her gait [26]. By considering all these aspects, our current study focused on how the unsupervised migration technique is used in basketball training to determine the player's activity.

## 3. Methods

### 3.1. Data Processing

Using the dataset and the intended meaning, an appropriate data model is created. There is a training set of data being examined, and each attribute has a class label assigned to it. After randomly selecting samples from the training dataset and dividing them by the training dataset, it is customary to apply directed learning to classify the data. Supervised learning is used when the data analysis knows exactly which class is in the lead when it comes to the training samples. Otherwise, it is called “unsupervised learning,” which is just another name for clustering. The decision tree is put through its paces using data analysis. The other data analysis is no longer relevant if the decision tree cannot guarantee its accuracy. Data analysis on decision trees can be done in a variety of ways. Classification accuracy is measured by looking at the percentage of data that was correctly categorized using a decision tree classification method. As a rule, we use well-known information rules as a benchmark and evaluate the model's predictions against the standard. If there is a huge disparity in the comparison results, the accuracy rate will be lower when the difference is greater. For this study, the data was obtained from NBA combined draught measurements.

### 3.2. SVM

Support Vector Machine (SVM) seems to be a kind of classifier with a supervisor that finds the best split with both respondents' different classes. The classifier is defined by SVM based on the training data. The classifier provides the framework for the classification judgments. Based just on basis functions, the classifier is intended to split input data into different classes. Many SVM classifiers could also classify objects into two categories, but a multilevel classification method could also be used if necessary. The classifier can be thought of as a function-described line. One such line is chosen to be as far away from all the data points as possible, reducing the impact of noise density. The SVM algorithm's task is to find the best possible margin hyperplane that considers the high data margin with both classes. Hyperparameters seem to be for collecting semantic data from basketball audio/video parameters for whose values control the learning system and determine the value systems of design variables that a learning algorithm learns. The training of the classification algorithm based on the equipment is used for measurement. As a result of this, the learning process and model parameters have been obtained.

A new multimodal approach for collecting semantic data from basketball audio and video will be first segmented and classified at a low level using the visual, movement, and audio and video elements retrieved from it. The basketball audio/video knowledge base is also used to detect important events. Together, visuals and motion are important in video. Shot and image boundary detection algorithms use prediction information, which is accompanied by analysis and classification. Audio essential sounds are collections of distinct audio sounds associated with linguistic events, and audio essential sound recognition is done using a deep learning classification method based on the Support Vector Machine (SVM) algorithm. The placements of likely lexical events, such as “foul” with “shoot just at basket,” are then discovered with additional technical experience by analyzing multimodal input. Furthermore, the algorithm generates a video description, and the testing results show that the proposed method is efficient.

To identify shot boundaries in the first stage, we utilize the differential between the statistical features of surrounding frames, *F*_*h*_, as that of the feature, which also is described as follows:

(1) $$\begin{array}{c} F_{h}=\frac{\sum_{i=0}^{P}\left|D_{n}\left(i\right)-D_{n-1}\left(\left(i\right)\right.\right|}{\text{Width}\cdot \text{Heigth}}\;>S_{g}, \end{array}$$

where *P* denotes the number of colour histogram bins,  *D*_*n* _ and *D*_*n*−1_ signify the color histograms of clips *n* with *n* − 1, respectively,  Width · Height signifies the pixel counts in every frame, and *S*_*g*_ denotes the thresholds for recognizing a single maximum activity in a series of *F*_*h* _ discontinuities values.

(2) $$\begin{array}{c} {\text{RFD}}_{n}=\left\{\begin{array}{cc} \frac{{\text{WF}}_{n-1}}{{\text{Hi}}_{n-1}}\;, & \text{for }I-\text{frame},\\ \frac{{\text{Ip}}_{n}}{{\text{WF}}_{n}}, & \text{for }b\text{ frame},\\ \frac{\left|{\text{WF}}_{n}-{\text{Hk}}_{n}\right|}{{\text{Hi}}_{n}}, & \text{for }H\text{ frame}, \end{array}\right. \end{array}$$

where Ip, WF, Hk, and Hi of equation (2) are the HBs for intracoded, forward forecasted, backward predicted, and bidirectionally predicted frames, correspondingly, and *n* is the frame size. We changed the Resource Description Framework(RFD) by (1) establishing a *b*-frame RFD formulation to provide more precise providing excellent when the boundary occurs at *I*-frames, and (2) modifying the H-frame RFD calculation to reduce false alerts if WF_*n*_ and HK_*n*_ are both much more than Bin. Examine the following frame construction. Analyze the frame construction.

(3) $$\begin{array}{c} {\text{DHBC}}_{n}=\left\{\begin{array}{cc} \left({\text{Hk}}_{n+1}-{\text{WF}}_{n+1}\right)\leq 0,\text{ for }I\text{ frame},\\ 1, & \text{otherwise, for }H\text{ frame}, \end{array}\right. \end{array}$$

(4) $$\begin{array}{c} dmx_{i}=b_{1}x_{i}+b_{2}y_{i}+b_{3}, \end{array}$$

where *dmx*_*i*_ and *dmy*_*i*_ of equation (4) are the areolation components for a specific bounding box.

*b*_*i*_'s are the linear parameters that we term interpolation linear parameters, while *x*_*i*_ and *y*_*i* _ are the locations of the HB's centroid.

We describe the row vector *r*_*i*_=(*x*_*i*_, *y*_*i*_, 1). Then, for all blocks that are not tagged as outliers, the coordinate matrix *C* is created by vertically concatenating the row vectors *r*_*i* _. *M* is the number of macroblocks that are not tagged as outliers, so *R* is a *M*  × 3 matrix. The vectors *U*_*x*_ and *U*_*y*_ are created by adding all of the *dmx*_*i*_ with *dmy*_*i* _ for the HBs that are not recognized as outliers. Finally, the interpolation linear parameters *b*_*x*_=(*b*_1_, *b*_2_, *b*_3_)^*T*^ with *b*_*y*_=(*b*_4_, *b*_5_, *b*_6_)^*T*^ are combined together. We may write *U*_*x*_=*Rb*_*x*_ and  *U*_*y*_=*Rb*_*y*_ based on these equations, which are then computed for *b*_*x*_ and *b*_*y*_ using *R*'s formation matrix as in the following:

(5) $$\begin{array}{c} b_{x}={\left(R^{T}R\right)}^{-1}R^{T}U_{x},\\ b_{y}={\left(R^{T}R\right)}^{-1}R^{T}U_{y}. \end{array}$$

Horizontal Motion Of Camera (HDC), Vertical Motion Of Camera (VDC), and Zoom Camera (ZDC). The above features are defined as in the following equations:

(6) $$\begin{array}{c} \text{HDC}=\frac{\sum_{i=0}^{M}b_{3i}}{M}, \end{array}$$

(7) $$\begin{array}{c} \text{VDC}=\frac{\sum_{i=0}^{M}b_{6i}}{M}, \end{array}$$

(8) $$\begin{array}{c} \text{ZDC}=\sum_{i=0}^{M}\frac{b_{1i}+b_{5i}}{2}, \end{array}$$

where *M* is the total number of frames in the picture.

Cepstral frequency coefficient is calculated as follows:

(9) $$\begin{array}{c} \text{Freq}\left(f\right)=3595\times \;\log_{10}\left(1+\frac{f}{700}\right), \end{array}$$

where Freq(*f*) is the standard frequency scale's logarithmic scale. The frequency scale covers and the frequency range of *R*_*n*_=0–30050 Hz 0–30050 Hz and also has a constant frequency spacing are represented as follows:

(10) $$\begin{array}{c} R_{n}=\sqrt{\frac{2}{k}}\sum_{k=1}^{k=1}\left(\log\;S_{k}\right)\;\cos\left[\left(nk-0.5\right)\frac{\pi }{k}\right],\;n=1,2,\ldots ,M. \end{array}$$

The changes of the voice signal are measured by the energy. With audio recordings *A*_*n*_, where *n* = 1, 2, ..., *M*: the energy is determined as the log of a signal energy as in the following:

(11) $$\begin{array}{c} V=\log\sum_{n=1}^{M}A_{n}^{2}. \end{array}$$

The above-mentioned methods are used in the proposed model (Figure 1).

The proposed model explains how the migrating method is used in basketball training in the form of audio and video. Level 1 and Level 2 are identified in the playing surface view. Fast playing and slow playing surface view and penalty come under Level 2. In another category, out of playing or fast playing medium surface view has been considered.

Figure 2 represents frequency analysis for audio and video basketball training using the SVM algorithm. Once the audio and video signal is given as input to the observation vector, then it undergoes training and testing. The outcome from the data preparation evaluates the probabilities of SVM algorithm.

## 4. Results and Discussion

In this section, the results have been analyzed using the proposed algorithm. For the given model, frequency has been classified for level 1 and level 2 categories. Support Vector Machine (SVM) is a classifier with a supervisor that finds the best split with different respondent classes. The classifier is defined by SVM based on the training data. The classifier provides a framework for the classification judgments. Based on the defined functions, the classifier is intended to split input data into different classes. Many classifiers like SVM could also classify objects into two categories. A multilevel classification method could also be used if necessary. The classifier can be thought of as a function-described line. One such line is chosen to be as far away from all data points as possible, reducing the impact of noise density. The SVM algorithm's task is to find its best possible margin hyperplane that considers the high data margin with both classes.

In Figure 3, it is observed that the support vector machine technique performs data-level classification of various data kinds, filters them, and removes errors in conjunction with the judgment function inside this procedure; second, it integrates the characteristics of various sorts of athletes. Different types of arrays have illustrations, and their data fit is further differentiated. Furthermore, the amount of deep learning methods used in the analysis of different football training arrays differs, and they will differ from one type to the next (Table 1).

The frequency of classification for level 1 and level 2 categories is increased. Thereby, the frequency regions corresponding to the edges are highlighted. It is typically used to calculate the estimated absolute luminance size at every point in a grayscale image. Support Vector Machine (SVM) is still a kind of classification model with a supervisor that finds the best separation among respondents in different classes. The classifier is defined by SVM based on the training data. The classifier defines the scope of the classification decision-making. Based just on basis functions, the classifier is intended to distribute input data into different classes.

In Figure 4, by combining several neural network analysis methodologies and selected superresolution elements to construct a successful relationship between pedestrian detection and different dynamic performances, the variables that have a stronger effect on the sports training procedure may be identified. It has been discovered that sports have such low-resolution difficulty during training. They set up a number of control trials to finalize the multifunctional application of various facts and information (Table 2).

In Figure 5, the performance analysis for vertical basketball using the deep learning method is observed. The application of SVM algorithms in sports and discovered that the different dialectical approach based on the deep learning method was used for data processing in the training data analysis link of football sports and discovered that this method seems to have more benefits (Table 3).

The method of basketball players accepting various styles of training programmers was introduced, and the particle swarm technique for optimization assessment was developed, along with an SVM algorithm based on the Randomization matrix. In Figure 6, the results demonstrate that the algorithm can help solve the problem of sports players' gait recognition while fluid movement, although it does so at the expense of partial recognition accuracy (Table 4).

In Figure 7, the results suggest that the algorithm can alleviate the problem of sports athletes' gait recognition during fluid movement, but it does so at the expense of incomplete recognition accuracy. The suggested deep learning method for dislocation gait identification is based on ant colony and particle swarm algorithms to enhance recognition accuracy. It has a high level of precision and can recognize the athlete's stride during the training process. This can identify the heel joint's rotational motion and the training effect.

Table 5 indicates the performance analysis of basketball training using the deep learning method. This reveals that the algorithm has high precision, which helps to determine the training effects.

In this proposed system, a high accuracy rate and precision and recall assessing the classification performance are used. We achieved an accuracy of recall of 0.9874 and a precision of 0.9978. A classification model for a basketball ref's hand motion indicators was implemented. We acquired a recognition performance of 0.9874 and an accuracy of 0.9978 while using the SVM classification.

The failure rate of training and body movement recognition within-group using the deep learning method is lower than in the group using the Support Vector Machine (SVM) algorithm, according to the results obtained by the three training methods (Table 6). The training system made use of an SVM method and data mining. The accuracy of experimental data shows an integration trend as training times are increased. When such several test times are reached, the transformation in error extent is very small, and the data accuracy could indeed be achieved in the best result for the SVM method, at 98.74%, compared to other CNN and NN algorithms.

## 5. Conclusion

In China, the sports industry has been enhanced well, but the efficiency of sports training needs to be developed. This paper focused on the training system of basketball to solve the issue of high-efficiency use of data and intelligent acquisition in sports training systems. When compared to the latest research results, the proposed method used in this research can achieve the effects of sports training. The experimental results indicate that sports training based on an unsupervised migration support vector machine (SVM) algorithm can analyze the model construction of video and audio and help athletes during training. The evaluation of the impact of different postures on sports athletes needs to be further studied. The proposed model is compared with the existing system, and it is observed that the proposed system reaches 98.74% more accuracy than other algorithms. For future research, it is highly suggested to implement the integration of machine learning with sensor techniques for managing basketball training. As a further extension, the players can be allowed to wear smart clothes to monitor their movements for further analysis.

## Figures and Tables

**Figure 1:** Overall architecture.

**Figure 2:** Frequency analysis for audio/video basketball using SVM algorithm.

**Figure 3:** Frequencies of classification for level 1 and level 2 categories.

**Figure 4:** Performance analysis for the height of basketball using deep learning.

**Figure 5:** SVM algorithm using performance analysis for vertical of basketball using deep learning method.

**Figure 6:** SVM algorithm using performance analysis for hand (width) and agility then sprint of basketball in the deep learning method.

**Figure 7:** SVM algorithm using overall performance analysis for basketball training in deep learning method.

**Table 1:** Frequencies of classification for level 1 and level 2 categories result.

Categories	Frequencies of classification (%)
Playing surface view	96.8
Flight view	99.9
Others	94.1
Fast playing surface view	93.6
Slow playing surface view	84.3
More than four fouls (penalty)	95.9
In fast playing medium surface view	89.7
Out of playing (or) close-up surface view	86.5

**Table 2:** Performance analysis for the height of basketball using deep learning result.

	Height (no shoes)	Height (with shoes)	Wingspan	Standing reach
Count	61.00	61.00	61.00	61.00
Mean	77.84	79.11	82.89	102.49
Std	3.42	3.40	3.71	4.98
Min	68.25	69.50	74.00	88.50
25%	75.75	77.00	81.00	100.00
50%	78.25	79.25	82.50	102.00
75%	80.25	81.50	86.50	106.50
Max	85.25	86.25	91.75	112.50

**Table 3:** SVM algorithm using performance analysis for vertical of basketball using deep learning method result.

	Vertical (max)	Vertical (max reach)	Vertical (no step)
Count	49.00	49.00	49.00
Mean	35.70	138.08	30.35
Std	3.77	4.29	3.54
Min	28.00	126.50	22.50
25%	33.50	135.00	27.50
50%	35.50	138.00	30.50
75%	38.00	141.00	32.50
Max	44.00	147.00	37.50

**Table 4:** SVM algorithm using performance analysis for hand (width) and agility then sprint of basketball using deep learning method result.

	Hand (width)	Agility	Sprint
Count	61.00	49.00	48.00
Mean	9.04	11.28	3.31
Std	1.46	0.57	0.13
Min	−1.00	10.26	3.12
25%	8.75	10.81	3.20
50%	9.25	11.25	3.26
75%	9.50	11.65	3.40

**Table 5:** Overall performance analysis for basketball training in deep learning method result.

Performance	Ground truth	Recall (%)	Precision (%)
Foul	30	97.4	97.7
Shot at the basket	50	96.8	91.3

**Table 6:** Comparison analysis for the start of the art method.

Performance	CNN algorithm	NN algorithm	SVM algorithm
Ground truth	28	27	30
Recall (%)	91.2	90.98	98.3
Precision (%)	94.2	92.49	99.1
Overall accuracy	92.43	91.45	98.74

## Data Availability

The data used to support the findings of this study are available from the corresponding author upon request.
